The article "NOD1 and NOD2 Are Potential Therapeutic Targets for Cancer Immunotherapy" was retracted in 2023. Reasons: signs of a paper mill; suspected computer-generated content; unreliable results or conclusions; concerns about the data.

# NOD1 and NOD2 Are Potential Therapeutic Targets for Cancer Immunotherapy

**DOI:** 10.1155/2022/2271788

**Published:** 2022-10-10

**Authors:** Dongjie Wang

**Affiliations:** Department of Pharmacy, Affiliated Cancer Hospital of Zhengzhou University and Henan Cancer Hospital, Zhengzhou, Henan 450003, China

## Abstract

The nucleotide oligomerization domain (NOD)-like receptors (NLRs) are a group of intracellular proteins that are essential for controlling the host's innate immune response. The cytosolic nucleotide binding oligomerization domains 1 and 2 receptors (NOD1 and NOD2) are the most widely investigated NLRs. As pattern recognition receptors (PRRs), NOD1 and NOD2 may recognize and bind endogenous damage associated molecular patterns (DAMPs) and external pathogenic associated molecular patterns (PAMPs), directing the activation of inflammatory caspases through engaging the adaptor protein RIP2, which further activates the NF-*κ*B and mitogen-activated protein kinase (MAPK) signaling pathways, thereby mediating host innate immunity and regulating the adaptive immunity. Previous research has identified NOD1 and NOD2 as key players in inflammatory disease and host-microbial defense. Despite numerous studies claiming that NOD1 and NOD2 are linked to tumorigenesis and tumor development, it is still unclear whether NOD1 and NOD2 act as cancer's friends or foes. In this review, we focus on concluding the current research progress on the role of NOD1 and NOD2 in a variety of cancers and discussing the potential reasons for the contradicting role of NOD1 and NOD2 in cancers. This review may help better understand the role of NOD1 and NOD2 in cancer and shed light on NOD1 and NOD2 as potential therapeutic targets for tumor immunotherapy.

## 1. Introduction

Innate immunity is crucial for resisting internal and external environmental stimuli and maintaining immune homeostasis. Innate immunity functions by nonspecifically identifying endogenous and exogenous risk factors via pattern recognition receptors (PPRs) [1]. TLRs and NLRs are important components of PRRs. TLRs are mainly found on the cell membrane, whereas NLRs are found primarily in the cytoplasm [2]. Although TLRs have been extensively studied for their role in multiple cancers [3, 4], increasing evidence suggests that NLRs, particularly, NOD1 and NOD2, have a close relationship with cancer cell proliferation, invasion, metastasis, and tumor angiogenesis. Due to the few reviews on the effect and mechanism of NOD1 and NOD2 in cancer, we will summarize the structural features of NLRs, including NOD1 and NOD2, as well as their role in carcinogenesis and tumor growth in this review.

## 2. The Discovery of NLRs and Their Structural Characteristics

NLRs were discovered at the end of the twentieth century. Initially, researchers discovered a type of protein in humans with a similar structure and physiological function to plant disease resistance receptors known as nucleotide binding-leucine rich repeats (NB-LRRs) [5]. Because of the similar capacity of initiating apoptosis after recognizing and binding the invading pathogens, “that type of proteins” in humans was named NLRs after NB-LRR. NLRs are encoded by NATCH genes, and NACHT domains include receptor neuronal apoptosis inhibitor protein (NAIP), telomerase associated protein 1 (TP1), MHC class II transcription activator (CIITA), and prosphora anserine incompatibility locus protein (HET-E) [4].

In humans, 22 different NLR types have been identified, compared to 33 different NLR types in mice [6, 7] (see Table 1). NLRs are extensively distributed in the cytoplasm, and this class of receptors typically consists of three parts: binding nucleotide oligomerization domain (NOD) in the middle segment, N-terminal regulatory domain, and C-terminal leucine repeats (LRRs). The two conservative domains LRRs and NOD are frequently present in the currently recognized NLRs [8]. The N-terminal domain is where NLRs differ most from one another [9, 10]; the N-terminal domains that have been discovered thus far include the acidic transactivation domain (AA), pyrin domain (PYD), caspase recruitment domain (CARD), death effector domain (DED), and baculovirus inhibitor repeat domain (BIR). Based on variations in the N-terminal domain, NLRs are classified into five subclasses: NLRA, NLRB, NLRC, NLRP, and NLRX. LRRs recognize and bind PAMPs and DAMPs, and when the ligand binds to LRRs, the NOD domain with natural ATPase activity self-oligomerizes and transfers the signal to the N-terminal domain, which subsequently connects with downstream signal molecules and initiates immunological response [8].

## 3. Structure of NOD1 and NOD2 and the Classic Activation Pathway

NOD1 and NOD2 are important members of the NLRs and also play a significant role in innate immunity. They were first identified as microbial detectors more than ten years ago.

Human chromosome 7p14-15 contains the gene that encodes the NOD1 receptor, while 16q12 houses the gene that encodes NOD2. NOD1 and NOD2, also known as NLRC1/CARD4 and NLPC2/CARD15, are found on many different types of cells, including macrophages, dendritic cells (DCs), Paneth cells, keratinocytes, and epithelial cells. While NOD1 is widely expressed in immune effector cells and lamina propria immune cells [11], NOD2 is mostly found in innate immune cells such as monocyte macrophages and dendritic cells, as well as epithelial cells of the lung, breast, kidney, and intestine [12]. Although NOD1 and NOD2 have the same structural formula of C-LRRs-NOD-CARD-N, NOD1 and NOD2 have different CARD domain numbers at the N-terminus when compared structurally with NOD1 having one while NOD2 having two [13] (see Figure 1).

The primary peptidoglycan (PGN) found in bacterial cell walls functions as both a natural agonist for NOD1 and NOD2 receptors. Bacterial particles that invade cells can break down into PGN, which triggers NOD1 and NOD2 directly. PGN can be injected into cells by extracellular bacteria using the type III transport system T3SS and the type IV transport system T4SS. In the meantime, peptide transporters-mediated transmembrane activity allows extracellular PGN to also enter host cells. PGN breakdown products, ie-DAP (*γ*-D-glu-mDAP) and muramyl dipeptide (MDP), have been shown to preferentially activate NOD1 and NOD2 receptors [14] (see Figure 2). Recognizing and combining PGN is a well-known NOD1 and NOD2 activation pathway. Nevertheless, when the PGN was recognized and bound to the LRRs, the activity of NOD1 and NOD2 was restored. Following self-oligomerization of the NOD domain, the signal was sent to the CARD domain at the N terminus, which was subsequently bound to the downstream serine-threonine kinase RIP2 signal protein through CARD-CARD contact, therefore activating the type I interferon, MAPK, and NF-*κ*B signaling pathways [15] (see Figure 3).

NOD1 binding to RIP2 enabled it to bind TNF receptor-associated factor 3 (TRAF3), which consequently activated TANK-binding kinase 1 (TBK1) and IkappaB kinase epsilon (IKK*ε*).

NOD1/TRAF3 signaling then promotes the expression of IFN regulatory factor 7 (IRF7), interferon beta (IFN), and interferon-stimulated gene factor 3 (ISGF3), which could contribute to host defense against *Helicobacter pylori*. NOD2 activation led to the signaling-dependent activation of the mitochondrial antiviral signaling (MAVS) protein, which in turn stimulated the MAVS-IRF3-IFN*β* pathway for host defense against viral infection [15, 16].

The activation of NOD1 and NOD2 receptors in antigen-presenting cells (APCs) boosts T cell function and strengthens the adaptive immune response [4]. Moreover, NOD1 and NOD2 also played a key role in sustaining T cell activation and proliferation, whereas deletion of NOD1 and NOD2 promotes T cells for activation-induced cell death upon antigen exposure16.

## 4. NOD1 and NOD2 in Cancer

Human NOD1 and NOD2 receptors were not identified until the 20th century [11, 17, 18].

As PPRs, NOD1 and NOD2 have a simple structure that enables them to broadly recognize harmful chemicals and trigger an immediate immune response.

As scavengers, NOD1 and NOD2 receptors act by determining the function of pathogenic substances, which makes it possible to effectively remove risk factors endangering the host. NOD1 and NOD2 receptors can recognize and clean the internal and external pathogenic substances based on their structures.

In contrast to TLRs dispersed on the cell membrane, protein misfolding in the cell can be one of the DAMPs to activate NOD1 and NOD2 receptors in the cytoplasm and begin appropriate immunological responses, which will terminate and remove aberrant cells in time to preserve immunoenvironmental homeostasis. Previous research suggested that NOD1 and NOD2 have an antibacterial role by detecting and combining bacterial PGN [19]. Numerous studies have also revealed that genetic polymorphisms in NOD1 and NOD2 are linked to a higher risk of developing Crohn's disease [20]. Further studies revealed that NOD1 and NOD2 are linked to the occurrence and development of malignancies, in addition to their antivirus and anti-infection function [21]. By detecting gene mutations and protein misfolding in cells, NOD1 and NOD2 can function as checkpoints to limit the unchecked proliferation of abnormal cells, eliminate faulty cells by accelerating the apoptotic process, and reduce the formation of malignancies. However, some studies have indicated that the expression of NOD1 and NOD2 in tumors may reduce the effectiveness of treatment and aid in the growth of tumors. Therefore, based on the advancement of this field's research, we will describe the function of NOD1 and NOD2 in cancer here (see Table 2).

### 4.1. The Role of NOD1 in Tumorigenesis and Development

#### 4.1.1. Oral cancer

Gao et al. found that cigarette smoke extract (CSE) could inhibit NOD1 expression in human oral mucosal epithelial cells and that ie-DAP (NOD1 agonist) could reverse the CSE-mediated inhibition effect on NOD1 but downregulate IL-6, IL-8, TNF-, and IFN- in Leuk-1 cells, thereby greatly reducing the damage caused by smoking on oral squamous cells [45].

#### 4.1.2. Thyroid cancer

Bai et al. discovered that enhanced NOD1 expression is associated with a better prognosis in thyroid cancer patients. Furthermore, as compared to normal epithelial cells NTHY-ORI 3-1, NOD1 expression was dramatically enhanced in papillary thyroid cancer (PTC) cell lines such as TPC-1, BCPAP, and KTC-1. NOD1 activation enhanced PTC cell death via caspase-3 and caspase-9 pathways mediated by RIP2/TAK1 and MAPK pathways, whereas NOD1 depletion boosted PTC cell growth in vitro [23].

#### 4.1.3. Head and Neck Squamous Cell Carcinoma (HNSCC)

However, other studies showed that NOD1 rather than NOD2 was strongly expressed and connected to the higher production of IL-8 in head and HNSCC tissues compared to noncancerous matched tissue (NCMT). Inhibiting IL-8 with siRNA can reduce the expression of NOD1 and RIP2 in HNSCC cell lines such as SCC4, SCC9, and SCC25, which suppress the tumor development and improve survival rates [24].

#### 4.1.4. Esophageal Squamous Cell Carcinoma (ESCC)

Fusobacterium nucleatum (F. nucleatum) found in the oral cavity is associated with poor prognosis in patients with ESCC. It has been reported that F. nucleatum activated the NF-*κ*B pathway via the NOD1/RIPK2 pathway to promote tumor growth [25].

#### 4.1.5. Breast Cancer

Da Silva Correia revealed for the first time that NOD1 mediated carcinogenesis and tumor formation in a breast cancer model [26]. Their research discovered that NOD1 overexpression in the TriDAP-induced estrogen-sensitive cell line MCF-7 can inhibit tumor development, but NOD1 deficiency in MCF-7 cells accelerates tumor growth and increases estrogen-dependent tumor cell proliferation due to an inability to process NOD1-mediated TNF*α*-induced apoptosis with IL-8 upregulation.

#### 4.1.6. Gastric Cancer

Loss of NOD1 increases the inflammatory and damage responses in gastric epithelial cells and macrophages exposed to *Helicobacter pylori*, raising the possibility that NOD1 exerts its checkpoint function by modifying macrophages and preserving microbial persistence [27].

#### 4.1.7. Hepatocellular Carcinoma (HCC)

It has also been shown that NOD1 expression was decreased in HCC tissues compared to corresponding noncancerous liver tissues. NOD1 also increased hepatocellular carcinoma HCC chemosensitivity to sorafenib or 5-FU therapy by decreasing the SRC-MAPK signaling pathway and inhibited HCC cancer cell growth in vitro and in vivo [28]. Evodiamine, one of the key components obtained from Evodiae, was recently found to exert antihepatocellular carcinoma activity by increasing apoptosis by inhibiting NOD1/NF-*κ*B/MAPK signaling [29].

#### 4.1.8. Colorectal Cancer (CRC)

Yang et al. found that overexpression of the proteasome subunit alpha type-7 (PSMA7) was related to inhibition of NOD1 expression in CRC. PSMA7 activation in HCT116 cells hindered NOD1-mediated apoptosis and NF-*κ*B activation, whereas PSMA7 depletion restored NOD1 function and thus suppressed tumor development [22]. Chen et al. discovered that systemic NOD1 deletion accelerated the growth of colon cancers in colitis-associated and Apc tumor suppressor-related colon cancer models. NOD1 deficiency affects the intestinal epithelial cell barrier, leading to increased surface epithelial apoptosis.

AOM/DSS therapy enhanced intestinal permeability, which is related to epithelial cell proliferation, as well as the elevation of inflammatory cytokine production such as IL-6, IL-1, and TNF-*α*. Gut microbiota depletion with antibiotics decreased tumor formation in NOD1-deficient mice, emphasizing a relationship between the gut bacteria and the NOD1 signaling pathway in the control of inflammation-mediated colon cancer [30]. In contrast to Yang and Chen's results [29], Jiang revealed that highly expressed NOD1 in CRC patients is adversely linked with survival rate. They discovered that NOD1 activation increases CRC cell adhesion, migration, and metastasis via the MAPK pathway [31]. Furthermore, NOD1 maintained myeloid-derived suppressor cell (MDSC) immunosuppressive function in CRC by boosting MDSC cell proliferation and modifying their immunosuppressive ability via arginase-1 activity, which subsequently promoted tumor development [32].

#### 4.1.9. Prostate Cancer

Porphyromonas gingivalis is an oral keystone pathogen that causes severe periodontitis by interfering with the host's immunological homeostasis. Furthermore, it has been shown that PD-L1 was increased via the NOD1/NOD2 pathway in prostate cancer cells following infection with Porphyromonas gingivalis, indicating that chronic inflammation can promote tumor metastasis by changing the tumor microenvironment [33].

#### 4.1.10. Cervical Cancer

NOD1 expression steadily reduced throughout the development of cervical neoplasia to cervical cancer caused by HPV16 exposure. Since HPV16-positive cervical cancer cells were more likely to undergo apoptosis when NOD1 was activated, this suggested that NOD1-mediated apoptosis may help to prevent cervical cancer [34]. In contrast to Liu's result [34], NOD1 was shown to be significantly expressed in cervical squamous cell carcinoma (CSCC), and overexpression of NOD1 increased proliferation, invasion, and migration of CSCC cell lines by activating NF-*κ*B and ERK signaling pathways and increasing IL-8 production [35–37].

#### 4.1.11. Ovarian Cancer

According to Shen's research [36], serous ovarian cancer is resistant to taxol through the NOD1/RIPK2/NF-*κ*B inflammatory pathway, and NOD1/RIP2 promotes the growth of ovarian cancer by turning on NF-B signaling. However, they did not investigate if the effect is related to the microbiota in the ovary and the permeability of the ovarian wall, which might be disturbed by NOD1 expression [37].

### 4.2. The Role of NOD2 in Tumorigenesis and Development

#### 4.2.1. NOD2 in Mice Xenograft Tumor Model

In 2001, two groups of scientists from the United States and France reported comparable study findings in the same issue of nature [46, 47]. They discovered that the NOD2 gene mutation was linked to Crohn's disease (CD). Following that, several research studies discovered that NOD2 gene mutation increased the risk of ulcerative colitis (UC) [48, 49], whereas CD and UC were precancerous lesions to colon cancer [50]. However, an epidemiology research including 40,000 participants indicated that NOD2 polymorphism may not be the predominant risk factor for gastrointestinal disorders, although the NOD2 relationship with gastrointestinal cancer cannot be fully ruled out [51]. Furthermore, Daillère et al. discovered that *Enterococcus* hirae and Barnesiella intestinihominis, which are suppressed by NOD2 in the intestine and colon, had an antitumor impact as an adjuvant for cyclophosphamide therapy in MCA205 sarcoma-bearing mice. Their research suggests that the NOD2 receptor functions as an immunological checkpoint in colorectal cancer. Overexpression of the NOD2 can result in a “sterile environment” in the colorectal area. However, the anti-infection activity of NOD2 decreases the anticancer impact of cyclophosphamide, whereas NOD2 deletion can restore the efficacy of chemotherapy [38].

However, it has been revealed that the NlpC/p60 peptidoglycan hydrolase SagA promotes anti-PD-L1 antitumor efficacy via NOD2 in melanoma mice models, indicating that the microbiome is required for NOD2 activity as a cancer checkpoint [39]. Tumor cell-derived microparticles (T-MP) are natural biomaterials that transmit innate signals via NOD2. T-MPs were mostly taken up by intestinal epithelial cells (IECs), where they could activate NOD2 and its downstream MAPK and NF-*κ*B, inhibiting the formation of B16 melanoma and CT26 colon cancer in mice. These revealed that NOD2 activity as a tumor suppressor is linked to gut mucosal immunity [40].

#### 4.2.2. Lung Cancer

Researchers discovered that inhibiting NOD2 improved the chemotherapeutic sensitization of nonsmall-cell lung cancer (NSCLC) to paclitaxel in Lewis lung carcinoma (LLC) tumor-bearing mice [41].

#### 4.2.3. Hepatocellular Carcinoma (HCC)

NOD2 can prevent HCC induced by a high-fat diet (HFD) through STAT3 and MAPK signaling by decreasing steroid production and neutrophil and macrophage infiltration, which contributes to cell proliferation prevention [42]. It was discovered that NOD2 expression was entirely deleted or significantly downregulated in HCC tissues, and it was directly associated with advanced HCC stages. In vivo, NOD2 deletion enhanced carcinogenesis in mice treated with N-nitrosodiethylamine (DEN) and carbon tetrachloride (CCL4), as well as tumor development in xenograft HCC models. NOD2 activation inhibited tumor growth, colony formation, and HCC cell invasion. Moreover, NOD2 exerted an antitumor effect via stimulating the adenosine 5′-monophosphate-activated protein kinase (AMPK) signaling pathway by interacting with the AMPK-LKB1 complex, resulting in autophagy-mediated HCC cell apoptosis and enhanced HCC cell sensitivity to sorafenib, lenvatinib, and 5-FU treatment [43, 44].

#### 4.2.4. Endometrial Cancer (EnC)

Tripartite motif-containing 22 (TRIM22) expression was decreased in EnC tissues compared to neighboring normal tissues. While TRIM22 stimulation inhibited EnC cell migratory, invasive, proliferative, and cell cycle activities via binding NOD2 [44].

### 4.3. Can NOD1 and NOD2 Be Promising Therapeutic Targets?

At present, there is no immunomodulator targeting the NOD1 receptor that has been on the market or in clinical trials, although the specific NOD1 inhibitor ML130 (Nodinitib-1) is only used in lab research. In addition, mifamurtide has been developed as a NOD2 agonist for osteosarcoma by IDM pharmaceutical company. Based on the structure of MDP, mifamurtide was designed to activate NOD2 in macrophage and dendritic cells in order to enhance the antigen presentation to T cells which further contributes to prevent osteosarcoma progression (see Figure 4).

However, the role of NOD1 and NOD2 in cancer is complicated, indicating that more studies in this field are necessary. It has been found that NOD1 activation contributes to tumor suppression mainly through RIP2/TAK1/MAPK pathway-mediated apoptosis in oral cancer [45], thyroid cancer [23], breast cancer [26], and GC 27, whereas NOD1 overexpression is associated with tumor development with decreased chemotherapy sensitivity but enhanced immunosuppression in HNSCC 24, ESCC25, prostate cancer [33], and ovarian cancer [36]. Based on those studies, we examined the conflicting roles of NOD1 in HCC [28, 29], CRC [22, 30–32], and cervical cancer [34, 35] and found that NOD1-regulated apoptotic activation is a common feature in tumor suppression, whereas NOD1-mediated immunosuppression is another comparable characteristics in NOD1-promoted malignancy which has been described by several studies [31, 32].

Excessive apoptosis in innate immune cells has been revealed to be a primary source of considerable immunosuppression [52], which suggests that reduced apoptosis might occur when immunosuppression is downregulated, but the immunosuppression generated by epithelial cell apoptosis is yet unknown. Guo et al. [29] discovered that inhibiting NOD1 in HepG2 and SMMC-7721 with evodiamine might enhance apoptosis in these cells, although they did not examine the expression of PD-L1 and other checkpoint markers in these cells. Taken together, NOD1-mediated apoptosis and NOD1-mediated immunosuppression may be linked, although the fundamental mechanism requires additional investigation.

The interaction with the gut commensal microbiota is now the primary study area for NOD2 in cancer. According to several studies, NOD2 worked in concert with gut bacteria or bacterial components such as SagA and T-MPs to increase the effectiveness of PD-L1 in cancer immunotherapy [39]. However, another team discovered that NOD2 inhibition will increase the chemotherapeutic sensitivity of lung cancer metastases through inhibition of NOD2 alone had little effect on suppressing tumor development 48. Furthermore, the intestinal barrier was not affected by the experimental stimulation in their study, suggesting that there is a lack of interaction between intestinal bacteria and NOD2 further dampens NOD2 capacity of suppressing cancer proliferation and attributing to decreased chemotherapy sensitivity.

Similar findings have been shown in HCC research where NOD2 inhibited the spontaneous HCC when the interaction between NOD2 and tumor microenvironment including tissue microbiome was intact [42, 43]. It is reported that NOD2 limited microbes-mediated immunomodulator in CTX-treated cancer; however, they only showed apoptosis data instead of tumor data in NOD2 knockout mice treated with bacterial oral gavage, which lack the direct evidence to show that NOD2 is a checkpoint for CTX therapy [38].

Taken together, NOD1 and NOD2 could be potential therapeutic targets for cancer with further investigation into their mechanism in different types of cancers.

## 5. Conclusions

NOD1 and NOD2 are PRR members that play an important role in immune homeostasis. Numerous studies have recently revealed that NOD1 and NOD2 have a close relationship with a variety of cancers via controlling proliferation, altering immunosurveillance, and interacting with tissue bacteria, including intestinal commensal intestinal microflora. Moreover, additional research into the mechanisms of NOD1 and NOD2 in cancers would shed light on the innate immunity-cancer relationship and provide intriguing targets for immunotherapy.

## Figures and Tables

**Figure 1:** NOD1 and NOD2 structure diagrams. The common structure of NOD1 and NOD2 is LRRs-NOD-CARD. NOD1 has 953 amino acids and one CARD domain, whereas NOD2 has 1040 amino acids and two CARD domains.

**Figure 2:** Structure of bacterial peptidoglycan (PGN) in Gram-positive and Gram-negative bacteria. As a NOD1 selective agonist, ie-DAP is made up of D-*γ*-Glu and mDAP, which is derived mostly from Gram-negative bacteria. While MDP, as a natural NOD2 agonist, is derived from both Gram-positive and Gram-negative bacteria with a structure composed of MurNAc, L-Ala, and D-*γ*-Glu.

**Figure 3:** NOD1 and NOD2 activation in response to PGN. Initially, NOD1 and NOD2 were suppressed by LRRs binding to NOD. Once PNG was recognized and bound to LRRs, NOD1 and NOD2 are activated by binding RIP2 and TAK1, which further activated the MAPK, NF-*κ*B, and type I interferon signaling pathways.

**Figure 4:** Potential mechanism of NOD1 and NOD2 in cancer. NOD1 exerts antitumor efficacy via apoptosis, whereas uncontrolled apoptosis-mediated by NOD1 would induce immunosuppression regulated by NOD1 and hence promotes tumor proliferation. Furthermore, the antitumor function of NOD2 is dependent on identifying and binding bacteria and their derivatives, when this connection is inadequate, NOD2 contributes to chronic inflammation and promotes cancer.

**Table 1:** NLRs in humans and mice.

NLR Family	N Terminus	NLR members (HGNC symbols)		Aliases
		Human	Mouse	
NLRA	AA	CIITA		NLRA; MHC2TA; C2TA
			Cllta	Nlra; MHC2TA; C2TA C2TA

NLRB	BID	NAIP		NLRB1; BIRC1; CLR5.1
			Naip1	Birc1a
			Naip2	Birc1b
			Naip3	Birc1c
			Naip4	Birc1d
			Naip5	Birc1e
			Naip6	Birc1f
			Naip7	Birc1g

NLRC	CARD	NOD1		NLRC1; CARD4; CLR7.1
			NOD1	Nlrc1; Card4
		NOD2		NLRC2; CARD15; CD; BLAU; IBD1; PSORAS1; CLR16.3
			NOD2	Nlrc2; Card15
		NLRC3		NOD3; CLR16.2
			NLRC3	CLR16.2
		NLRC4		CARD12; CLAN; CLR2.1; IPAF
			NLRC4	Card12; CLAN; Ipaf
		NLRC5		NOD27; CLR16.1

NLRP	PYD	NLRP1		NALP1; DEFCAP; NAC; CARD7; CLR17.1
			Nlrp1a	NALP1a
			Nlrp1b	NALP1b
			Nlrp1c	NALP1c
		NLRP2		NALP2; PYPAF2; NBS1; PAN1; CLR19.9
			Nlrp2	Pypaf2; Nbs1; Pan1
		NLRP3		CIAS1; PYPAF1; Cryopyrin; NALP3; CLR1.1
			Nlrp3	Cias1; Pypaf1; Cryopyrin; Nalp3; Mmig1
		NLRP4		NALP4; PYPAF4; PAN2; RNH2; CLR19.5
			Nlrp4a	Nalp4a; Nalp-eta; Nalp9D
			Nlrp4b	Nalp4b; Nalp-gamma; Nalp9E
			Nlrp4c	Nalp4c; Nalp-alpha; Rnh2
			Nlrp4d	Nalp4d; Nalp-beta
			Nlrp4e	Nalp4e; Nalp-epsilon
			Nlrp4f	Nalp4f; Nalp-kappa; Nalp9F
			Nlrp4g	Nalp4g
		NLRP5		NALP5; PYPAF8; MATER; PAN11; CLR19.8
			Nlrp5	Mater; Op1
		NLRP6		NALP6; PYPAF5; PANS; CLR11.4
			Nlrp6	
		NLRP7		NALP7; PYPAF3; NOD12; PAN7; CLR19.4
		NLRP8		NALP8; PAN4; NOD16; CLR19.2
		NLRP9		NALP9; NOD6; PAN12; CLR19.1
			Nlrp9a	Nalp9a; Nalp-theta
			Nlrp9b	Nalp9b; Nalp-delta
			Nlrp9c	Nalp9c; Nalp-zeta
		NRLP10		NALP10; PAN5; NOD8; PYNOD; CLR11.1
			Nlrp10	Nalp10; Pynod
		NRLP11		NALP11; PYPAF6; NOD17; PAN10; CLR19.6
		NRLP12		NALP12; PYPAF7; Monarch1; RNO2; PAN6; CLR19.3
			Nlrp12	Nalp12
		NRLP13		NALP13; NOD14; PAN13; CLR19.7
		NRLP14		NALP14; NOD5; PAN8; CLR11.2
			Nlrp14	Nalp14; Nalp-iota; GC- LRR
NLRX1	DED			NOD9; CLR11.3

**Table 2:** Summary of reported associations between NOD1/NOD2 and cancer progression.

NLR member	Cancer	Research topic	Findings	Reference
NOD1	Oral cancer	The effect of cigarette smoke (CSE) extract on human oral squamous cells	NOD1 protects the oral squamous cell from damage caused by smoking by decreasing IL-6, IL-8, TNF-*α,* and IFN-*γ* expression	[22]
	Thyroid cancer	NOD1 in papillary thyroid cancer (PTC)	NOD1 promoted PTC cell apoptosis via caspase-3/9 through RIP2/TAK1/MAPK pathway	[23]
	Head and neck squamous cell carcinoma (HNSCC)	IL-8 and NOD1 in HNSCC	IL-8 synergized with NOD1 promotes HNSCC by the CXCR1/2 signaling pathway	[24]
	Esophageal squamous cell carcinoma (ESCC)	Effect of Fusobacterium nucleatum on ESCC	Fusobacterium nucleatum promotes ESCC development by activation of the NOD1/RIPK2/ NF-*κ*B pathway	[25]
	Breast cancer	NOD1 in estrogen-sensitive cell breast cancer	NOD1 depletion in MCF-7 cells promotes tumor growth due to dysfunction of TNF*α*-induced apoptosis regulated by NOD1	[26]
	Gastric cancer	Effect of Helicobacter pylori on gastric epithelial cells and macrophages	NOD1 may modulate immune homeostasis by regulating macrophage and microbial persistence	[27]
	Hepatocellular carcinoma (HCC)	The role of NOD1 in Hepatocellular carcinoma	NOD1 enhanced the chemosensitivity and proliferation of HCC by suppressing the SRC-MAPK signaling pathway in vitro and in vivo	[28]
		Effect of evodiamine on HCC	Evodiamine induces apoptosis in vitro by suppressing NOD1/NF-*κ*B/MAPK pathway	[29]
	Colorectal cancer (CCR)	Mechanism of PSMA7 in CCR	NOD1 suppresses PSMA7-mediated CCR development by promoting apoptosis	[22]
		Interaction between NOD2 and commensal bacteria in CRC	NOD1 combined with intestinal commensal bacteria contribute to the suppression of CRC development in vitro and in vivo	[30]
		Effect of NOD1 on CRC metastasis	NOD1 is highly expressed in human CRC tissues; activation of NOD1 cell promote HT29 adhesion, migration, and metastasis by the MAPK pathway	[31]
		The immunosuppressive function of NOD1 in CRC	NOD1 promotes MDSCs proliferation and accelerates tumor progression in CRC	[32]
	Prostate cancer	Effect of PD-L1 on prostate cancer infected with *Porphyromonas gingivalis*	NOD1/2 promotes PD-L1 expression upon *Porphyromonas gingivalis* infection, thus, promotes tumor metastasis	[33]
	Cervical cancer	Association between NOD1 and invasive squamous cell carcinoma (ISCC)	NOD1 augments the apoptosis of HPV16-positive cervical cancer cells	[34]
		Role of NOD1 in cervical squamous cell carcinoma (CSCC)	NOD1 promoted CSCC proliferation, invasion, and migration via IL-8 and NF-*κ*B/ERK pathway	[35]
	Ovarian cancer	Mechanism of Taxol resistance on serous ovarian cancer	Activation of the NOD1/RIPK2/NF-*κ*B pathway promotes chemotherapy resistance to ovarian cancer	[36]
		Mechanism of NOD1 in ovarian cancer	Activation of the NOD1/RIP2/ NF-*κ*B pathway promotes ovarian cancer progression	[37]
NOD2	MCA205 sarcoma-bearing mice model	Mechanism of bacterial species involved in immunosurveillance during cyclophosphamide (CTX) treatment	NOD2 interferes with the adjuvant effect of *Enterococcus hirae* and *Barnesiella intestinihominis* for CTX treatment in xenograft mice model	[38]
	Melanoma xenograft mice model	Molecular mechanisms of the gut microbiome on host response to PD-L1 therapy	SagA promotes antitumor efficacy of PD-L1 therapy via NOD2 activation	[39]
	B16 melanoma and CT26 colon xenograft mice model	Investigation of the mechanism of antitumor vaccination based on gut mucosal immunity	T-MPs taken up by IEC suppress the tumor growth via NOD2/MAPK/NF-*κ*B pathway	[40]
	Lung cancer	Role of NOD2 in paclitaxel-treated lung cancer	NOD2 inhibition increased the NSCLC sensitization to paclitaxel	[41]
	Hepatocellular carcinoma (HCC)	The role of NOD2 in obesity-dependent HCC	NOD2 prevents HFD -induced HCC via STAT3/MAPK signaling	[42]
		NOD2 in HCC	NOD2 correlated with poor prognosis of HCC; Loss of NOD2 accelerates spontaneous HCC growth; NOD2 bind with AMPK enhances chemotherapy efficiency of HCC	[43]
	Endometrial cancer (EnC)	Role of TRIM22 in EnC	NOD2 synergized with TRIM22 to suppress EnC proliferation and metastasis	[44]

## Data Availability

The dataset can be obtained from the author upon request.
